# Clinical Study of Sentinel Lymph Node Detection to Evaluate Pelvic Lymph Node Metastasis to Determine the Prognosis of Patients with Early Cervical Cancer

**DOI:** 10.1155/2022/8394049

**Published:** 2022-03-23

**Authors:** Peipei Li, Shuai Feng, Guodong Zhou, Lu Zhang, Xiugui Sheng, Dapeng Li

**Affiliations:** ^1^Department of Gynecologic Oncology, Shandong Cancer Hospital and Institute, Shandong First Medical University and Shandong Academy of Medical Sciences, Jinan 250117, China; ^2^Department of Maternity, Jinan Maternal and Child Health Hospital Affiliated to Shandong First Medical University, Jinan 250001, China; ^3^National Cancer Center, National Clinical Research Center for Cancer and Cancer Hospital & Shenzhen Hospital Chinese Academy of Medical Sciences, Peking Union Medical College, Shenzhen, Guangdong 518116, China

## Abstract

**Objective:**

Lymph node status is one of the most important prognostic factors for uterine cervical cancer. Sentinel lymph node (SLN) biopsy has emerged as a potential alternative to systematic lymphadenectomy for the lymph node mapping in such patients. However, the SLN metastasis detection via SLN biopsy in early-stage cervical cancer remains controversial. The current study is aimed at investigating the feasibility and accuracy of combined tracer method for localization of SLN in initial stages of cervical cancer and to evaluate the clinical value of SLN biopsy in replacing pelvic lymph node resection.

**Methods:**

We retrospectively reviewed 348 cases who were admitted to the Department of Gynecologic Oncology, Shandong Provincial Cancer Hospital, China, between February 2003 and June 2018 with FIGO stage IA2 to IIA2 cervical cancer and undergone through SLN biopsy. Methylthioninium chloride was injected in combination with ^99m^technetium-labeled sulfur colloid prior to surgery to these patients. SLNs were identified intraoperatively, excised, and subsequently submitted to fast frozen section. The detection rates, accuracy, sensitivity, coincidence rate, false negative rate, and negative predictive values of these cases were estimated, and the follow-up outcomes were carefully observed. Chi squared test or Fisher's exact test was employed for a comparison of the categorical variables. Univariate and multivariate Cox proportional hazard models were used for estimation of relationships between overall survival (OS) and disease-free survival (DFS) and prognostic factors.

**Results:**

The total detection rate of SLN was 97.1% (338/348), and identification of bilateral SLN was successful in 237 patients (70.1%). The patient's tumor size, FIGO stage, lymph node metastasis, and depth of invasion had statistically significant differences in SLN detection rates. The detection rate had inverse relation with tumors size (>4 cm), invasive depth > 2/3, lymph node positive, late staging, and preoperative radiotherapy. 117 positive SLNs were detected in 73 patients. The negative predictive value, sensitivity, false negative rate, and coincidence rate and were 97.7%, 92.4%, 7.6%, and 95.4%, respectively. In patients whose tumor size were ≦ 4 cm, the false negative rate was 4.55% (2/44), whereas it was 0 in patients with tumor size≦2 cm. The respective 1, 3, and 5-year OS was 100%, 94.8%, and 91.8%, respectively, whereas DFS rate for 1, 3, and 5 years was 96.7%, 92%, and 89.6%, respectively. The lymph node was positive, tumor size, the depth of invasion, and staging were statistically different from the recurrence rate and survival rate of patients (*p* < 0.05). When tumor metastasis exceeded SLN, the recurrence rate was significantly increased, and survival rate is significantly reduced (*p* < 0.05, *p* < 0.01, *p* < 0.05, respectively).

**Conclusions:**

The identification of SLN combined with ^99m^technetium-labeled sulfur colloid and methylthioninium chloride has a good accuracy and is safe for the assessment of the status of pelvic nodes in patients with initial stage cervical cancer. Nuclide as a tracer has low dependence on objective conditions and doctors' technology and has a good detection rate. In our study, we believe that SLN biopsy is feasible when the tumor is ≦ 4 cm. Large scale clinical trials are required in China expand the sample size and validate the results of this study.

## 1. Introduction

Cervical cancer prevalence has increased in China in recent years. At present, the staging system of the International Federation of Gynaecology and Obstetrics (FIGO) has included lymph node metastasis as the most notable predictive factor for survival and recurrence in cervical cancer patients who have been surgically treated [1–3]. The early-stage patients manifested pelvic lymph node metastasis at a rate of about 10-34% [4–7], nearly two-thirds of lymphatic metastasis patients suffered from the complications due to unnecessary dissection of the pelvic lymph node. These complications include immune function and postoperative neurological damage, lymphocele, infection, urination dysfunction, double lower limbs, and perineum edema complications, affecting the patient's life quality seriously.

Imaging studies such as CT, MR, and PET have low sensitivity to lymph node metastasis. The sentinel lymph node biopsy (SLNB) can predict the preoperative condition of regional lymph node metastasis. If SLN shows no metastasis, full lymph node dissection can be omitted, to shorten the operation time, reduce the surgical complications, and provide personalized therapy for patients. SLNB has been used as the standard of care for surgical staging in a number of cancers including breast cancer, skin cancer, and vulvar cancer, and it is also widely employed in endometrial cancer and cervical cancer. In 2015, the National Comprehensive Cancer Network (NCCN) included and recommended SLNB in its guidelines for stage IA2-IIA1cervical cancer patients [8]. However, the SLN metastasis detection via SLN biopsy in early-stage cervical cancer remains controversial.

In this study, we investigated the feasibility, accuracy, and limitations of SLN biopsy for cervical cancer in its early stages by looking at topographic localization of SLN and patterns of lymphatic dissemination to pelvic lymph nodes. We investigated the feasibility and accuracy of combined tracer method for localization of SLN in initial stages of cervical cancer and evaluated the clinical value of SLN biopsy in replacing pelvic lymph node resection.

## 2. Materials and Methods

### 2.1. Data Source and Study Population

Enrolled women included those referred for abdominal (laparotomic or laparoscopic) radical hysterectomy for initial cervical cancer (2009 FIGO stageIA2 toIIA2) between November 2002 and June 2018. Patients undergo intraoperative SLN detection followed by radical hysterectomy and systematic pelvic lymphadenectomy. Para-aortic lymph node sampling was carried out in 28 of these enrolled individuals. Assessment of the tumor location, size, and cranial extent was made in all patients by a combination of abdominal ultrasound and magnetic resonance imaging.

### 2.2. The SLN Biopsy Technique

Using the combined tracer method, 0.5 ml of ^99m^Tc-labeled sulfur colloid and 1 ml of methylene blue were injected 3, 6, 9, and 12 o'clock positions into the mucosa of the cervix, 6-18 h before surgery. Intraoperative visual recognition of blue-stained lymph nodes was considered SLN. A handheld gamma probe (Neoprobe, neo2000TM: AR-MED, Ltd.) was employed for their detection, and the presacral area, pelvic sidewall, and para-aortic lymph beds were completely scanned. The existence of radioactive hot nodes measuring >5-fold above the background level was the characteristic feature used to identify SLNs. After localization, the SLNs were excised in situ and sent to a rapid frozen pathological examination, followed by pelvic lymphadenectomy or radical hysterectomy combined with abdominal para-aortic lymphadenectomy or absence thereof. The resected tissues were sent for standard pathological evaluation, and the presence of micrometastases (≤2 mm) in the lymph node sections was detected using immunohistochemical methods. The above pathological examinations were completed by at least two senior pathologists, and the results were checked. According to the results of the routine pathological examinations, postoperative adjuvant therapy was performed on patients having risk factors for recurrence.

### 2.3. Statistical Analysis

The chi squared test or Fisher's exact test was employed for a comparison of the categorical variables. Significance was defined as a *p* value <0.05. SPSS version 22.0 (SPSS Inc, Chicago, IL, USA) was used for all analyses. To investigate relationships between DFS or OS and prognostic factors, investigators employed univariate and multivariate Cox proportional hazard models, and the 2-tailed *p* value <0.05 was considered statistically significant.

### 2.4. Follow-Up

Survival, relapse, or death statistics were obtained from outpatient or by calling the patient. The date of diagnosis was used to calculate overall survival. On the date of the last follow-up, the surviving patients were censored. Within two years of treatment, patients were followed up every three months, once every six to twelve months during the next three years, and once every five years. Patients who lost to follow-up were omitted from the follow-up results analysis.

## 3. Results

### 3.1. The Relation between Clinicopathological Features and Lymph Node Metastasis

The total 348 patients had a median age of 44 years (range 22–77 years). Among these 348 patients, 89% were squamous cell carcinoma patients, 7% were adenocarcinoma patients, and 4% were other histological cancer type stage Ia2, Ib1, Ib2, IIa1, and IIa2 patients which accounted for 4.9%, 44.3%, 20.7%, 8.9%, and 21.2%, respectively. Their lymph node metastasis rates were 5.9%, 16.9%, 34.7%, 29%, and 32.4%, respectively. The lymph node metastasis rate was 37.7% (40/107) in patients with local tumor > 4 cm, 18.6% (45/2241) in ≦4 cm. 222 (range 1-16) positive lymph nodes were found in 85 cases (85/348, 24.4%); among them, patients with tumors >4 cm accounted for 60% (51/85). 88 para-aortic lymph nodes were excised from 28 individuals, and the metastatic rate amounted to 7.1% (2/28). Patients with IA2 or higher cancer stage, moderate to poor differentiation, >1/3 infiltration depth, and tumor size > 4 cm, and lymph node metastasis rate increased significantly (*p* < 0.01, *p* < 0.01, *p* < 0.01, and *p* < 0.01, respectively). Body mass index (BMI), histological type, and preoperative adjuvant therapy for lymph node metastasis were not significantly different. Besides, there was no correlation between BMI and the number of lymph nodes metastases.  Table 1 summarizes the patients characteristics.

### 3.2. SLN Detection Results

8010 lymph nodes, in total, were removed from 348 cases (mean = 23; range 6-47). There were 1277 SLNs identified in the population of 338 patients, with the estimated median per patient being 3.8. SLNs were successfully identified in 338 patients, as shown in Figure 1. In 73 patients, 117 SLNs were found to be positive. The obturator (49%) was found to be the most common site for SLN detection, with 75.4% (255/338) patients having it, followed by the external iliac (31%) with 55.6% (188/338) patients having it. We also found 101 SLNs within the internal iliac, 36 in the cardinal ligament, 89 in the common iliac, 27 in the parametric region, and 3 in the presacral regions. In the para-aortic area, no SLN was discovered. The pelvic lymph node localization area was basically the same as SLNs.

Among 10 patients who identified SLN unsuccessfully, of which 6(60%) were positive for lymph nodes, patients with tumors > 4 cm accounted for 80% (8/10), patients with IB2 or higher accounted for 90% (9/10), and those with invasive depth≧2/3 accounted for 80% (8/10) as shown in Table 2.

We used a combination of methylthioninium chloride and ^99m^technetium-labeled sulfur colloid as tracers to obtain a SLN detection rate of 97.1% (338/348), and the detection rate of ^99m^technetium-labeled sulfur colloid tracer SLN was higher than the detection rate of methylene blue (96.83% vs. 74.3%, *p* < 0.01). 146 patients (42%) underwent neoadjuvant chemotherapy and/or brachytherapy before the surgical procedure. Among them,109 patients underwent concurrent chemoradiotherapy, and the detection rate was 96.33%. 24 patients received only radiotherapy, and their detection rate was 95.83%. 13 patients received only chemotherapy, and their detection rate was 92.3%. Preoperative chemotherapy and local radiotherapy did not influence the rate of detection of SLN.

In 237(70.1%) of 338 patients, bilateral pelvic SLNs were detected, and 72.2% of them had tumors with a size ≤ 4 cm.  Table 3 shows the interrelation between the rate of SLN detection and various clinical attributes. In patients with IB1 or higher stage, tumors > 4 cm, lymph node positive, and invasive depth > 1/3, the total rate of detection of SLN was significantly reduced (*p* < 0.05, *p* < 0.05, *p* < 0.05, *p* < 0.05, respectively), but BMI, cell differentiation, and histology did not affect SLN detection rate. It can also be seen from the table that when the invasion depth was >2/3 and lymph node metastasis, the bilateral rate of detection of SLN is significantly reduced (*p* < 0.01 and *p* < 0.01, respectively) as shown in Table 3.

The respective percent values of sensitivity, coincidence rate, and negative predictive value were 92.4%, 95.4%, and 97.7%, respectively, and the false negative rate was 7.6% (6/79). 6 cases of false negative patients had lymph node metastasis. 66.7% (4/6) of these patients had tumor size > 4 cm, 50% (3/6) of these patients had IB2-IIA2 cancer stage, and 66.7% (4/6) of them invaded the outer 1/3 and the full layer. In patients whose tumor size was ≦2 cm, the patient's sensitivity, coincidence rate, and negative predictive value reached 100%, and the false negative rate was equivalent to 0. When tumor size was ≦ 4 cm, the sensitivity, coincidence rate, and negative predictive value were 95.5%, 99.2%, and 99%, respectively. The false negative rate raised to 4.17% (2/48). When the tumor size was >4 cm, the sensitivity, coincidence rate, and negative predictive value were 89.74%, 95.96%, and 93.75%, respectively, and the false negative rate was 10.26%. Results of immunohistochemical staining showed no isolated tumor cells (ITCs) or missed micrometastases (lesions < 2 mm) in SLNs.

### 3.3. Outcomes of Follow-Up

As of July 2018, the median follow-up time was 64 months (range, 1-171 months). 82 of 348 (23.56%) patients did not report for follow-up, leading to a rate of follow-up equivalent to 76.4%. The data analysis did not include the responses of the patients who lost to follow up. The remaining 266 patients were followed up, and there were a total of 24 (9%) cases recurrence at average months of 37 (13-144). 91.7% (21/23) cases occurred within 5 years after diagnosis. Among them, 6 patients had a recurrence in the pelvic cavity, 8 in the lung, 3 in the inguinal lymph nodes, 1 in the supraclavicular lymph nodes, 3 in the vaginal stump, and 1 in the para-aortic lymph node, In 1 case, the pelvic cavity and lungs were involved, and 1 case of pelvic and vaginal stump recurrence was observed. 17 patients died of tumor progression in the course of follow-up. The disease-free survival at 1, 3, and 5 years was 96.7%, 92%, and 89.6%, and actuarial overall survival was 100%, 94.8%, and 91.8%, respectively.

The relationship between recurrence and clinical pathological characteristics is shown in Table 4. Patients with positive lymph nodes, tumors > 4 cm, stage II cancer, lymph-vascular space invasion, and invasive depth > 1/3 muscle layer had significantly higher recurrence rates than other groups (*p* < 0.05). Contrarily, there was no considerable difference in recurrence rates among groups with various histological types, BMI, or degrees of differentiation. Tumor size, FIGO stage, depth of invasion, lymph node metastasis, and lymphatic vessel infiltration were found to be risk factors for 5-year OS and DFS in patients depicted by the univariate analysis (*p* < 0.05) (Table 5). Multivariate analysis revealed lymph node metastasis as an independent prognostic risk factor for patients with recurrence, DFS, and OS (*p* < 0.001) as shown in Table 6.

Based on lymph node metastasis, we categorized the patients into three groups: lymph node negative, the tumor only invades the first station lymph node (only SLN is positive), and the tumor invades more than two stations (SLN and non-SLN are positive). Prognosis analysis showed that the disease-free survival rate and recurrence rate between the three groups were significant statistically (*p* = 0, *p* < 0.001, respectively). When the lymph nodes were positive, the patient was more likely to relapse, especially when it goes beyond SLN, and the recurrence rate and disease-free survival rate increased significantly (*p* < 0.05). Among the three groups, the overall survival rate was not significant statistically, but was significantly reduced when tumors were transferred to lymph nodes other than the first station (*p* < 0.05) (in Table 7). Among 23 patients with recurrence and metastasis, we statistically analyzed the location of recurrence and metastasis and found that patients were prone to metastasis in the lungs. The lung metastases of these three groups were 27.3%, 25%, and 62.5%. When other pelvic lymph nodes were positive, the lung metastasis rate was significantly increased (after we have ruled out tumor size, depth of invasion, degree of differentiation, intravascular thrombosis, and staging of these risk factors).

## 4. Discussion

The latest edition of the National Comprehensive Cancer Network (NCCN) Practice Guide considers SLNB only for patients with stage I; although, it can be used in patients with tumor sizes < 4 cm, but SLN is best at <2 cm [9]. Many published studies demonstrate the feasibility of SLNB for cervical cancer [10–12], and there is currently some evidence that SLNB without lymph node resection have the same oncology results with reduced complications. In case of patients with stage IA/IB1/IIA1 cervical cancer, preliminary data from the randomized SENTICOL2 study comparing the morbidity of pelvic SLNB plus lymphadenectomy versus SLNB alone showed a considerable decrease in early postoperative neurologic deficits (7.8 vs. 20.6%) and surgical complications (1.4% vs. 51.5%) in the SLNB alone group [13]. Yahata et al. investigated the surgical complications and prognostic outcome in early-stage cervical cancer patients who underwent SLNB for trachelectomy or hysterectomy [14]. They discovered that operative time, blood loss, and the development of lymphangitis and lymphedema were considerably lower in patients who underwent SLNB than in patients who underwent matched pelvic lymphadenectomy, and it is assumed that the prognostic results are not different between the two groups. Their study, however, has drawbacks similar to Niikura et al. [15]. Particularly since it is not a randomized control trial, women who want to safeguard and conserve their fertility are also availing SLNB, with favorable obstetrical outcomes.

Lymph node metastasis is one of the most critical risk factors for the identification and prognosis of patients who require adjuvant chemoradiation treatment, according to the 2018 FIGO staging system for uterine cervical cancer. A normal lymphatic drainage pattern from the cervix to regional lymph nodes was described by Plentl and Friedman [16]. The regional lymph nodes include parametrial, para-aortic, and common iliac nodes [17], but the detection of the parametric node is rather difficult since it lies close to the cervix. According to several studies [18, 19], 80% of SLNs are found in pelvic tissues, with the external iliac being the most prevalent site for SLN detection. Our findings were identical to those reported, with the exception that the majority of SLNs (49%, 625/1277) were found in the obturator. Only 31% (396 of 1277) SLNs were found in the external iliac. A total of 29.9% of the 338 individuals in our study had unilateral pelvic SLNs. One plausible explanation is that SLN lymphatic drainage possibly occurs on one side of the pelvis. Previous research has also found similar results [20]. We believe that “SLN” is a functional and not an anatomical concept. The “skip metastasis” of the lymph node is relative in terms of anatomical location. When the first involved node is the second station lymph node of the cervix, its function is equivalent to a first station lymph node. The “skip metastasis” has important clinical significance for further clarifying the lymphatic drainage channel of the cervix and range of surgical resection. When the positive SLNs are located in common iliac area, the aortic lymph nodes should be dissected at the same time.

In our investigation, the SLN detection rate was 97.1%, and the sensitivity, coincidence rate, negative predictive value (NPV), and the false negative rate of the SLNs were 92.4 percent, 95.4 percent, 97.7%, and 7.6%, respectively. Sentinel lymph nodes (SLNs) have been shown to have an 89% detection rate and a 90% sensitivity rate in cervical cancer [21]. Pelvic lymph node status, invasion depth, tumor size, and FIGO stage are all factors that influence SLN detection rates, as suggested by our findings. The SLN detection rate was substantially greater in women without metastases than in women with metastases (*p* < 0.05), which is also in agreement with the published reports [22]. Furthermore, we discovered that the SLN detection rate was the substantially higher in-patient group belonging to stage I (*p* < 0.01), and that the SLN detection rate is 99% (284/287) in patients with a tumor size≦4 cm and 100% in patients with a tumor size of ≦ 2 cm. The procedures involving sentinel lymph node biopsy have better accuracy with small-sized tumors and in patients with bilaterally identified SLNs, as suggested by the published data to date [23, 24]. We believe that when the stage IB1 or above and the tumor is >4 cm, the optimal injection site (normal cervical tissue around the tumor) decreases or disappears, and there may be local tissue necrosis. When the lymph node metastasis rate is high, the metastatic lymph nodes block the lymphatic vessels, hindering the passage of the tracer and reducing the SLN detection rate. In addition, our study concluded that preoperative radiotherapy or chemotherapy did not affect the detection rate of SLN; however, no studies on this have been reported, which may be insufficient powered to draw accurate conclusions due to the limited number of cases we counted.

For lymphatic mapping in uterine and cervical cancers, the fluorescent dye indocyanine green (ICG) has been explored as an offlabel as an alternative to blue dye. ICG had a relatively tiny sample size, but it can minimize radiation exposure, cause no pain, and cost a lot less in comparison to other treatments involving radiation [25], but some objective conditions of ICG will affect the detection rate of SLN, such as patient BMI, timing and location of injection (submucosal injection and intramuscular injection), and identification equipment. In contrast, nuclide requirements for objective conditions are relatively low, the identification device of the radionuclide is relatively simple, the intraoperative radiation is low, preoperative injection time range is 4-20 hours, and we all can get better SLN imaging, detection rate, and negative prediction value. Moreover, we also find that BMI does not affect SLN detection rate, whereas Snyman [26] reported that women with a BMI≧30 achieved a detection rate that was considerably low in comparison to women having a BMI≦25 (*p*<0.05). High BMI was found to hamper the identification of bilateral sentinel nodes using indocyanine green or blue dye, in one retrospective analysis. The effect, however, was substantially stronger with blue dye alone than with ICG alone [27]. Some literature has reported similar results [28]. In our study, although the detection rate of nuclide was higher than methylene blue (74.3% vs. 96.8%), the combination of methylene blue and nuclide would give a better result. Furthermore, several hospitals in China and some other developing countries, for economic reasons, do not currently have the facilities or are qualified enough to furnish ICG and related equipment. Therefore, we believe that nuclide is less dependent on recognition equipment, physician level, preoperative injection time, and patient obesity, and combining nuclide and blue dye labeling is the best choice for tracing SLN in China or in economically underdeveloped areas and under limited doctor' injection and technical level.

For SLNB, the ability to acquire an accurate intraoperative diagnosis is rather critical. Lymph node metastasis has been documented in 15% to 20% of patients with early-stage cervical cancer (ESCC). If the preoperative imaging or intraoperative biopsy lymph node is negative in patients with ESCC (a tumor diameter of <4 cm and FIGO stage IA2, IB1, and IIA), the missed micrometastasis rate is only 0.08% [29], and pelvic lymphadenectomy is not generally considered as a requirement. Micrometastasis, according to some experts, is a major cause of postoperative recurrence and distant metastasis. The clinical stage is earlier, and the recurrence rate following radical surgery in cervical cancer patients without lymph node metastases is 10% to 15%, with tumor size and stage influencing the incidence [30]. Yahata et al. reported that as compared to the bisection along the longitudinal axis, the sensitivity of diagnosis is higher in 2 mm slices along the short axis [31]. Patients with endometrial cancer, cervical cancer, and colorectal cancer have been investigated by employing the one-step nucleic acid amplification (OSNA) technique, which identifies mRNA within metastatic lymph nodes [32–34], and the OSNA method has been used to detect the expression of human papillomavirus-E6 squamous cell carcinoma antigen or cytokeratin 19 in cervical cancer [33]. We also performed OSNA, and early results revealed that out of 36 involved, one patient was falsely positive, and one patient was falsely negative. OSNA in combination with intraoperative fast results in improved accuracy, which will be reported in future studies. It renders intraoperative lymph node metastasis identification easier and has the potential to make SLNB the gold standard for minimally invasive surgical procedures.

To circumvent the high FNR of SLNBs, Cormier et al. [35] proposed an SLN algorithm. It involves a side-specific evaluation and suggests lymphadenectomy on the side(s) when no SLNs are found, along with the resection of clinically enlarged lymph nodes, with a final NPV and sensitivity equivalent to 100%. Although predominantly SLN biopsy investigations have shown a detection rate of 95–100%, an NPV of 97–100%, and an FNR of 0–8% [36], there is still a debate due to the comparatively high FNR in patients having large cervical tumors [18, 21, 37]. We discovered that ten false-negative patients had an SLNB at an early stage of our SLN detection, and that 60% (6/10) of the top 50 patients who underwent sentinel lymph node biopsy failed to detect it; so, we believe that learning curve is a factor that influences SLN detection accuracy in SLNB. The skill level and training of the surgeon are key factor in SLNB, SAWAI, and other trials [38]. Doctors must undertake at least 10 sentinel lymph node biopsy procedures, and the detection rate of sentinel lymph nodes will grow by more than 90%, but the false negative rate will be greater than 5% before less than 30 sentinel lymph node biopsy operations. The false negative rate was found to be 0.08% in patients with tumors≦4 cm and no preoperative or intraoperative questionable nodes with bilateral negative SLNs after ultra staging, in a study of 46 trials involving 4130 individuals [29]. Yuan [19] and Wydra et al. [39] both found a similar pattern. A retrospective review by Kim et al. [40] found that SLN biopsy alone may be possible in early-stage cervical cancer, when the size of the tumor is less than 2 cm and lymph node metastasis is not suspected in image examination. Nevertheless, to ascertain whether or not SLN biopsy alone can be performed in early cervical cancer, large-scale prospective studies are required. The intrinsic false-negative rate of SLN biopsy in breast cancer patients was shown to be in the range of 4–10% [41, 42], and the recommendation by the American Society of Breast Surgeons suggest an 85% SLN detection rate with an FNR of 5% or less [43]. When the tumor size was 2 cm, the false negative rate was 0; when the tumor size was 4 cm, the sensitivity, coincidence rate, negative predictive value, and false negative rate were 92.2%, 97.4%, and 4.55% (2/44), respectively. As a result, we feel that sentinel lymph node biopsy can be used for the assessment of the status of pelvic lymph nodes when the tumor≦4 cm. Furthermore, we discovered a considerable rise in the false negative rate in lymph node metastatic patients (*p* < 0.01). According to Soergel [44], sentinel detection employing a combination of Tc-99mnanocolloid and ICG and or a mixed ICG-^99m^Tc-nanocolloid molecule may lower the sentinel method's false negative rate. In conclusion, the combined tracer approach, immunohistochemistry, and PCR-based molecular techniques for micrometastasis of lymph nodes can reduce the false-negative rate as much as feasible.

According to certain studies, using SLNB to treat early-stage cervical cancer is effective and safe, and it does not raise the risk of recurrence [14]. In previous randomized controlled trials comparing lymph node dissection to SLN biopsy only to for patients suffering from breast cancer, overall survival and disease-free survival were shown to be identical [45, 46]. According to our follow-up, FIGO stage, LVSI, lymph node metastases, and deep invasion are risk factors for the patient's recurrence rate and 5-year survival rate (all *p* < 0.05). Lymph node metastasis remained an independent predictive factor for lower overall survival rate and early cervical cancer disease-free survival (*p*≦0.001) as suggested by a multivariable analysis. A recent study compared recurrence-free survival in patients with stage IA/IB cervical cancer who had undergone pelvic lymph node dissection versus sentinel lymph node biopsy alone in patients with node-negative disease and found no difference among the groups in terms of overall survival and recurrence-free survival at 2 and 5 years [47]. Due to objective reasons, we did not compare lymph node dissection with SLN biopsy only for individuals suffering from early-stage cervical cancer, but further statistical analysis revealed that when the tumor invades the second station lymph node or more, the recurrence rate was significantly higher, and the survival rate was significantly lower than with SLN alone. If SLNB is not performed, the position when the lymph node was positive, and giving postoperative adjuvant therapy becomes difficult. By doing SLNB, it clearly show the location of positive lymph nodes. When tumor invasion exceeds SLN, considering more aggressive treatment after surgery, for example, radiation therapy has a wider extension field, a larger dose of radiation or more cycles of chemotherapy. Therefore, sentinel lymph node biopsy to guide postoperative treatment has important clinical significance for patient survival and recurrence rate. A number of evidences demonstrate the significance of carrying out a future multicenter trial. We anticipate the same promising outcomes for SLNB in patients suffering from cervical cancer.

## 5. Conclusions

SLNB has been used as the standard of care for surgical staging in several cancers, and the National Comprehensive Cancer Network (NCCN) included and recommended SLNB in its guidelines for stage I cervical cancer patients. However, the SLN metastasis detection via SLN biopsy in early-stage cervical cancer remains controversial. This study was aimed at investigating the feasibility and accuracy of the combined tracer method for localization of SLN in the initial stages of cervical cancer and to evaluate the clinical value of SLN biopsy in replacing pelvic lymph node resection. The size of the tumor, the extent of lymph node metastases, and the depth of invasion all play a role in the success rate of SLN identification. Based on our findings, we believe that sentinel lymph node biopsy is viable when the tumor≦4 cm in diameter. The use of nuclide and blue dyes as tracers has a low reliance on objective conditions and medical technology, and it has a high detection rate. The identification of SLN combined with ^99m^technetium-labeled sulfur colloid and methylthioninium chloride has a good accuracy and is safe for the assessment of the status of pelvic nodes in patients with initial stage cervical cancer. Furthermore, using sentinel lymph node biopsy to assess pelvic lymph node metastases to guide postoperative treatment has significant clinical implications for patient survival and recurrence rates. To properly validate the results of this study, large sample-sized clinical trial studies of SLNB in China are needed.

## Figures and Tables

**Figure 1:** Localization and status of pelvic nodes and SLNs (the picture is taken from the book “Clinical Gynecologic Oncology”).

**Table 1:** The relationship between clinicopathological features and lymph node metastasis.

Characteristics	No. of patients (%)		No. of patients with positive nodes(%)		*p*
Histology					
Squamous cell carcinoma	310	89%	77	24.8%	>0.05
Adenocarcinoma	24	7%	5	20.8%	>0.05
Else	14	4%	3	21.4%	
BMI					
≦25	228	65.5%	58	25.4%	>0.05
>25, ≦30	101	29%	25	24.8%	
>30	19	5.5%	2	10.5%	
FIGO stage					
Ia2	17	4.9%	1	5.9%	<0.01^a^
Ib1	154	44.3%	26	16.9%	
Ib2	72	20.7%	25	34.7%	<0.01^b^
IIa1	31	8.9%	9	29%	
IIa2	74	21.2%	24	32.4%	
Differentiation					
Grade I	67	19.2%	8	11.9%	<0.05^c^
Grade II	146	42%	45	30.8%	<0.05^d^
Grade III	135	38.8%	32	23.7%	
Invasion depth					
≤1/3	135	38.8%	20	14.8%	<0.01^e^
1/3-2/3	51	14.7%	7	13.7%	
>2/3	100	28.7%	26	26%	<0.01^f^
Whole cervix	62	17.8%	32	51.6%	
Tumor size (cm)					
≤4 cm	241	69.8%	45	18.6%	<0.01^∗^
>4 cm	107	30.2%	40	37.7%	
Preoperative radiotherapy					
Yes	133	38.2%	37	27.8%	>0.05
No	215	61.8%	48	22.3%	
Preoperative chemotherapy					
Yes	122	35.1%	35	28.7%	>0.05
No	226	64.9%	50	22.1%	

^a, c, e^ *p* value between each group, ^b^*p* value between stage I and stage II, ^d^*p* value between grade I and grade II, and ^f^*p* value between ≦ 2/3 and>2/3.

**Table 2:** Patients with unsuccessful SLN detection.

No.	Age	FIGO stage	BMI	Histology	Differentiation	Muscle depth of invasion	Tumor size (cm)	Metastatic nodes	Vessel invasion
1	52	Ib2	28.8	^∗^SCC	Grade II	>2/3	6	1	—
2	70	IIa	26.9	SCC	Grade II	Whole cervix	5	6	—
3	49	IIa	24.9	SCC	Grade I	1/3-2/3	4	1	—
4	55	IIa	27.2	SCC	Grade III	Whole cervix	4.5	1	—
5	57	Ib1	25	SCC	Grade II	>2/3	2.5	0	—
6	44	IIa	27.5	SCC	Grade III	Whole cervix	5	1	—
7	25	Ib2	23.1	SCC	Grade I	>2/3	5	0	+
8	46	Ib2	23.3	SCC	Grade I	1/3-2/3	6	0	—
9	44	Ib2	27.2	SCC	Grade II	>2/3	5	16	—
10	42	Ib2	27.9	^∗^Adeno	Grade I	>2/3	4.5	0	—

^∗^SCC: squamous cell carcinoma. ^∗^Adeno: adenocarcinoma.

**Table 3:** Relationship between clinical characteristics and SLN detection.

Characteristics	SLN detection			P1	P2
	Bilateral	Unilateral	None		
Histology					
Squamous cell carcinoma	210	91	9	>0.05	>0.05
Adenocarcinoma	17	6	1		
Else	10	4	0		
BMI (kg/m^2^)					
≦25	153	77	5	>0.05	>0.05
>25, ≦30	67	16	5		
>30	17	8	0		
FIGO stage					
Ia2	16	1	0	<0.05^g^	>0.05
Ib1	107	46	1		
Ib2	49	18	5	<0.01^h^	>0.05
IIa1	21	9	1		
IIa2	44	27	3		
Differentiation					
Grade I	52	13	2	>0.05	>0.05
Grade II	95	46	5		
Grade III	90	42	3		
Invasion depth					
≤1/3	104	31	0	<0.05^i^	<0.05^j^
1/3-2/3	39	10	2		
>2/3	58	37	5	≤0.05	<0.01^k^
Whole cervix	36	23	3		
Tumor size (cm)					
≤4 cm	171	64	2	<0.01^∗^	>0.05
>4 cm	66	37	8		
Lymph node metastasis					
Yes	39	40	6	<0.05^∗^	<0.01^∗^
No	198	61	4		
Preoperative radiotherapy					
Yes	75	42	5	>0.05	>0.05
No	162	59	5		
Preoperative chemotherapy					
Yes	82	46	5	>0.05	>0.05
No	155	55	5		

P1: *p* value of LN detection rate; P2: *p* value of SLN double-sided detection rate; ^g, i^*p* value between the total detection rates of each group; ^h^*p* value between the total detection rate of stage I and stage II, ^j^*p* value of bilateral detection rate between groups, and ^k^*p* value of double-sided detection rate between ≦ 2/3 and >2/3; ^∗^denotes statistically significant difference.

**Table 4:** The relationship between recurrence and clinical pathological characteristics.

Variable	Recurrence	No recurrence	*p* value
Histology			
Squamous cell carcinoma	21	219	>0.05
Adenocarcinoma	2	14	
Else	1	9	
LNM			
Yes	12	39	<0.01^∗^
No	12	203	
LVSI (yes)			
Yes	5	26	<0.05^∗^
No	19	216	
FIGO stage			
I	12	173	<0.01^∗^
II	12	69	
Differentiation			
Grade I	2	48	>0.05
Grade II	9	98	
Grade III	13	96	
Invasion depth			
≤1/3	9	97	<0.05^∗^
1/3-2/3	2	36	
>2/3	4	74	
Whole cervix	9	35	
Tumor size (cm)			
≤4 cm	12	159	<0.05^∗^
>4 cm	12	55	
BMI (kg/m^2^)			
≦25	14	159	>0.05
>25, ≦30	8	70	
>30	2	13	

LVSI: lymph-vascular space invasion; ^∗^denotes statistically significant difference.

**Table 5:** Univariable analyses for DFS and OS.

Variables	5-years OS				5-years DFS			
	Survival rates	HR	95%CI	*P*	Survival rates	HR	95%CI	*P*
Tumor diameter, mm								
≦2cm	100	2.7	(1.163,6.269)	<0.05^∗^	100	2.149	(1.087,4.248)	<0.05^∗^
>2cm,≤4cm	92.7				90.4			
>4cm	86.6				83.6			
BMI(kg/m^2^)								
≦25	91.8	1.242	(0.561,2.750)	>0.05	89.9	1.292	(0.678,2.461)	>0.05
>25,≦30	89.5				87.4			
>30	85.7				88.9			
Histology								
Squamous cell carcinoma	92.4	1.246	(0.544,2.856)	>0.05	89.5	1.289	(0.453,2.397)	>0.05
Adenocarcinoma	87.5			>0.05	87.5			>0.05
else	88.9				90.0			
LNM								
No	97.1	9.874	(3.478,28.032)	<0.001^∗^	94.5	4.209	(1.892,9.397)	<0.01^∗^
Yes	72.9				71.5			
LVSI								
No	93.4	3.223	(1.132,9.171)	<0.05^∗^	91.4	2.167	(0.803,5.848)	>0.05
Yes	77.6				72.6			
FIGO Stage								
Ia2	100	2.064	(1.203,3.540)	<0.01^∗^	100	1.471	(0.950,2.277)	<0.05^∗^
Ib1	94.9				91.7			
Ib2	92.5			0.010^∗^	90.4			>0.05
IIa1	84.2				83.0			
IIa2	82.4				81.8			
Differentiation								
Grade I	95.7	1.467	(0.735,2.927)	>0.05	95.8	1.801	(0.977,3.321)	0.05
Grade II	91.4				90.8			
Grade III	90.4				86.8			
Invasion Depth								
≤1/3	92.4	1.551	(1,2.405)	0.050^∗^	91.5	1.289	(0.904,1.840)	>0.05
1/3-2/3	100				96.7			
>2/3	94.8				93.5			
whole cervix	77.6				72.8			

**Table 6:** Multivariable analyses for DFS and OS.

Variables	5-year DFS			5-year OS		
	HR	95% CI	*p*	HR	95% CI	*p*
LNM (yes)	10.253	(1.708, 9.253)	0.001^∗^	15.977	(3.053, 26.138)	<0.01^∗^

^∗^denotes statistically significant difference.

**Table 7:** Relationship between sentinel lymph node metastasis and prognosis.

Variables	No. of patients	Recurrence rate	*P*	1-years OS	3-years OS	5-years OS	*P*	1-years DFS	3-years DFS	5-years DFS	*P*	OS			DFS		
												HR	95%CI	*P*	HR	95%CI	*P*
SLN(-) and LN(-)	211	5.2% (11/211)	0.000^∗^	1	95.40%	93.20%	>0.05	96.90%	92.30%	89.90%	<0.001∗			0.578			<0.001∗
SLN(+) and LN(-)	30	13.3% (4/30)	<0.05∗	1	96.30%	91.90%	<0.05∗	1	89.30%	81.00%	<0.01∗	0.963	(0.215, 4.303)	0.96	1.297	(0.492, 3.418)	>0.05
SLN(+) and LN(+)	20	40% (8/20)		1	91.70%	78.60%		88.50%	67.30%	43.60%		2.194	(0.491, 9.812)	0.304	5.267	(2.332, 11.89)	<0.001

## Data Availability

Data will be provided on request.

## References

[1] Pecorelli S. (2009). Revised FIGO staging for carcinoma of the vulva, cervix, and endometrium. *International Journal of Gynecology & Obstetrics*.

[2] Biewenga P., van der Velden J., Mol B. W. J. (2011). Prognostic model for survival in patients with early stage cervical cancer. *Cancer*.

[3] Macdonald O. K., Chen J., Dodson M., Lee C. M., Gaffney D. K. (2009). Prognostic significance of histology and positive lymph node involvement following radical hysterectomy in carcinoma of the cervix. *American Journal of Clinical Oncology*.

[4] Li X., Yin Y., Sheng X. (2015). Distribution pattern of lymph node metastases and its implication in individualized radiotherapeutic clinical target volume delineation of regional lymph nodes in patients with stage IA to IIA cervical cancer. *Radiation Oncology*.

[5] Fuchs J., Hamann M. F., Schulenburg F. (2013). Sentinel-Lymphknotenbiopsie beim Peniskarzinom. *Der Urologe*.

[6] Benedetti-Panici P., Maneschi F., Scambia G. (1996). Lymphatic spread of cervical cancer: an anatomical and pathological study based on 225 radical hysterectomies with systematic pelvic and aortic lymphadenectomy. *Gynecologic Oncology*.

[7] Fuller A. F., Elliott N., Kosloff C., Lewis J. L. (1982). Lymph node metastases from carcinoma of the cervix, stages IB and IIA: implications for prognosis and treatment. *Gynecologic Oncology*.

[8] Koh W.-J., Greer B. E., Abu-Rustum N. R. (2015). Cervical cancer, version 2.2015. *Journal of the National Comprehensive Cancer Network*.

[9] Wood D. E. (2015). National Comprehensive Cancer Network (NCCN) clinical practice guidelines for lung cancer screening. *Thoracic Surgery Clinics*.

[10] Bats A.-S., Mathevet P., Buenerd A. (2013). The sentinel node technique detects unexpected drainage pathways and allows nodal ultrastaging in early cervical cancer: insights from the multicenter prospective SENTICOL study. *Annals of Surgical Oncology*.

[11] Cibula D., Dusek J., Jarkovsky J. (2019). A prospective multicenter trial on sentinel lymph node biopsy in patients with early-stage cervical cancer (SENTIX). *Cancer*.

[12] Lecuru F. R., McCormack M., Hillemanns P. (2019). SENTICOL III: an international validation study of sentinel node biopsy in early cervical cancer. A GINECO, ENGOT, GCIG and multicenter study. *Cancer*.

[13] Mathevet P., Lécuru F., Uzan C. (2021). Sentinel lymph node biopsy and morbidity outcomes in early cervical cancer: results of a multicentre randomised trial (SENTICOL-2). *European Journal of Cancer*.

[14] Yahata H., Kobayashi H., Sonoda K. (2018). Prognostic outcome and complications of sentinel lymph node navigation surgery for early-stage cervical cancer. *International Journal of Clinical Oncology*.

[15] Niikura H., Okamoto S., Otsuki T. (2012). Prospective study of sentinel lymph node biopsy without further pelvic lymphadenectomy in patients with sentinel lymph node–negative cervical Cancer. *Cancer*.

[16] Plentl A. A., Friedman E. A. (1971). Lymphatic system of the female genitalia. The morphologic basis of oncologic diagnosis and therapy. *Major Problems in Obstetrics Gynecology*.

[17] Wiebe E., Denny L., Thomas G. (2012). Cancer of the cervix uteri. *International Journal of Gynecology & Obstetrics*.

[18] Fader A. N., Edwards R. P., Cost M. (2008). Sentinel lymph node biopsy in early-stage cervical cancer: utility of intraoperative versus postoperative assessment. *Gynecologic Oncology*.

[19] Kara P. P., Ayhan A., Caner B. (2008). Sentinel lymph node detection in early stage cervical cancer: a prospective study comparing preoperative lymphoscintigraphy, intraoperative gamma probe, and blue dye. *Annals of Nuclear Medicine*.

[20] O'Boyle J. D., Coleman R. L., Bernstein S. G., Lifshitz S., Muller C. Y., Miller D. S. (2000). Intraoperative lymphatic mapping in cervix cancer patients undergoing radical hysterectomy: a pilot study. *Gynecologic Oncology*.

[21] Kadkhodayan S., Hasanzadeh M., Treglia G. (2015). Sentinel node biopsy for lymph nodal staging of uterine cervix cancer: a systematic review and meta-analysis of the pertinent literature. *European Journal of Surgical Oncology*.

[22] Plante M., Renaud M. C., Têtu B., Harel F., Roy M. (2003). Laparoscopic sentinel node mapping in early-stage cervical cancer. *Gynecologic Oncology*.

[23] Yamashita T., Katayama H., Kato Y. (2009). Management of pelvic lymph nodes by sentinel node navigation surgery in the treatment of invasive cervical cancer. *Cancer*.

[24] Zarganis P., Kondi-Pafiti A., Arapantoni-Dadioti P. (2009). The sentinel node in cervical cancer patients: role of tumor size and invasion of lymphatic vascular space. *In Vivo*.

[25] Buda A., Crivellaro C., Elisei F. (2016). Impact of indocyanine green for sentinel lymph node mapping in early stage endometrial and cervical cancer: comparison with conventional radiotracer 99m Tc and/or blue dye. *Annals of Surgical Oncology*.

[26] Snyman L. C., Bryant E. P., Wethmar E. I. (2018). Use of a sentinel lymph node biopsy algorithm in a south African population of patients with cervical cancer and high prevalence of human immunodeficiency virus infection. *Cancer*.

[27] Eriksson A. G. Z., Montovano M., Beavis A. (2016). Impact of obesity on sentinel lymph node mapping in patients with newly diagnosed uterine cancer undergoing robotic surgery. *Annals of Surgical Oncology*.

[28] Salvo G., Ramirez P. T., Levenback C. F. (2017). Sensitivity and negative predictive value for sentinel lymph node biopsy in women with early-stage cervical cancer. *Gynecologic Oncology*.

[29] Tax C., Rovers M. M., de Graaf C., Zusterzeel P. L. M., Bekkers R. L. M. (2015). The sentinel node procedure in early stage cervical cancer, taking the next step; a diagnostic review. *Gynecologic Oncology*.

[30] Cibula D., Abu-Rustum N. R., Dusek L. (2012). Prognostic significance of low volume sentinel lymph node disease in early-stage cervical cancer. *Gynecologic Oncology*.

[31] Sonoda K., Yahata H., Okugawa K. (2018). Value of intraoperative cytological and pathological sentinel lymph node diagnosis in fertility-sparing trachelectomy for early-stage cervical cancer. *Oncology*.

[32] Kosťun J., Pešta M., Sláma J. (2019). One-step nucleic acid amplification vs ultrastaging in the detection of sentinel lymph node metastasis in endometrial cancer patients. *Journal of Surgical Oncology*.

[33] Okamoto S., Niikura H., Nakabayashi K. (2013). Detection of sentinel lymph node metastases in cervical cancer: assessment of KRT19 mRNA in the one-step nucleic acid amplification (OSNA) method. *Gynecologic Oncology*.

[34] Yamamoto H., Sekimoto M., Oya M. (2011). OSNA-based novel molecular testing for lymph node metastases in colorectal cancer patients: results from a multicenter clinical performance study in Japan. *Annals of Surgical Oncology*.

[35] Cormier B., Diaz J. P., Shih K. (2011). Establishing a sentinel lymph node mapping algorithm for the treatment of early cervical cancer. *Gynecologic Oncology*.

[36] Wuntakal R., Papadopoulos A. J., Montalto S. A., Perovic M., Coutts M., Devaja O. (2015). Location of sentinel lymph node in cervical carcinoma and factors associated with unilateral Detection. *Cancer*.

[37] Lukas R., Helena R., Jiri H. M., Martin H., Petr S. (2013). Current status of sentinel lymph node mapping in the management of cervical cancer. *Expert Review of Anticancer Therapy*.

[38] Sawai K., Nakajima H., Ohe S., Mizuta N., Sakaguchi K., Hachimine Y. (2002). Sentinel lymph node biopsy and low axillary node sampling for breast cancer. *Nihon Geka Gakkai Zasshi*.

[39] Wydra D., Sawicki S., Wojtylak S., Bandurski T., Emerich J. (2006). Sentinel node identification in cervical cancer patients undergoing transperitoneal radical hysterectomy: a study of 100 cases. *Cancer*.

[40] Kim J.-H., Kim D. Y., Suh D. S. (2018). The efficacy of sentinel lymph node mapping with indocyanine green in cervical cancer. *World Journal of Surgical Oncology*.

[41] Harlow S. P., Krag D. N., Julian T. B. (2005). Prerandomization surgical training for the National Surgical Adjuvant Breast and Bowel Project (NSABP) B-32 trial: a randomized phase III clinical trial to compare sentinel node resection to conventional axillary dissection in clinically node-negative breast cancer. *Annals of Surgery*.

[42] Veronesi U. (2003). The sentinel node and breast cancer. *Journal of British Surgery*.

[43] Lyman G. H., Giuliano A. E., Somerfield M. R. (2005). American Society of Clinical Oncology guideline recommendations for sentinel lymph node biopsy in early-stage breast cancer. *Journal of Clinical Oncology*.

[44] Soergel P., Kirschke J., Klapdor R., Derlin T., Hillemanns P., Hertel H. (2018). Sentinel lymphadenectomy in cervical cancer using near infrared fluorescence from indocyanine green combined with technetium-99m-nanocolloid. *Lasers in Surgery Medicine*.

[45] Krag D. N., Anderson S. J., Julian T. B. (2007). Technical outcomes of sentinel-lymph-node resection and conventional axillary-lymph-node dissection in patients with clinically node-negative breast cancer: results from the NSABP B-32 randomised phase III trial. *The Lancet Oncology*.

[46] Veronesi U., Paganelli G., Viale G. (2006). Sentinel-lymph-node biopsy as a staging procedure in breast cancer: update of a randomised controlled study. *The Lancet Oncology*.

[47] Lennox G. K., Covens A. (2017). Can sentinel lymph node biopsy replace pelvic lymphadenectomy for early cervical cancer?. *Gynecologic Oncology*.

